# SOFA Score in relation to Sepsis: Clinical Implications in Diagnosis, Treatment, and Prognostic Assessment

**DOI:** 10.1155/2022/7870434

**Published:** 2022-08-10

**Authors:** Changbo Liu, Shuzhen Suo, Liya Luo, Xixian Chen, Chunxiang Ling, Shixiong Cao

**Affiliations:** Department of Critical Medicine, The Fourth Affiliated Hospital of Guangzhou Medical University, Guangzhou, Guangdong, China

## Abstract

**Purpose:**

To analyze the clinical significance of the sequential organ failure assessment (SOFA) score in the diagnosis, treatment, and prognostic assessment of sepsis.

**Methods:**

140 patients with sepsis from January 2020 to January 2021 were selected as the observation group, and 40 healthy people were selected as the control group. The observation group was divided into mild group, severe group, and septic shock group by single blind grouping according to the condition of the disease, and they were also divided into survival group and death group according to the prognosis. Collect the fasting venous blood of the subjects in each group in the morning, compare the levels of total bilirubin (TBIL), blood creatinine (CR), and platelet count (PLT) in each group, and record and compare the patients' respiratory system oxygen partial pressure/inhaled oxygen concentration (po2/fio2), acute physiology and chronic health scoring system II (APACHE II), sequential organ failure assessment (sofa) score, q-SOFA score, and △SOFA score; Pearson analysis was used to analyze the correlation between SOFA score and other indicators; multivariate logistic regression was used to analyze the prognostic risk factors of patients with sepsis; receiver-operating characteristic curve (ROC) was used to analyze the value of SOFA score alone and in combination in the diagnosis, condition, and prognosis of sepsis.

**Results:**

There were significant differences in Apache II score, SOFA score, q-SOFA score map, po2/fio2, PLT, GCS, TBIL, and serum creatinine (SCR) between the control group and the observation group (*P* < 0.05). There were significant differences in Apache II score, SOFA score, q-SOFA score, mean arterial pressure (map) po2/fio2, PLT, Glasgow Coma Score (GCS), TBIL, SCR, and △SOFA score among patients in mild, severe, and septic shock groups (*P* < 0.05). There were significant differences in age, Apache II score, SOFA score, q-SOFA score, map, po2/fio2, PLT, GCS, TBIL, SCR, and △SOFA score between survival group and death group (*P* < 0.05). SOFA score and q-SOFA score were significantly positively correlated with TBIL and SCR and significantly negatively correlated with po2/fio2 and PLT; △SOFA score was significantly negatively correlated with TBIL and SCR and significantly positively correlated with map, po2/fio2, PLT, and GCS. Apache II score, SOFA score, and q-SOFA score were independent risk factors for sepsis patients, and △SOFA score, po2/fio2, and GCS score were protective factors (*P* < 0.05). ROC curve analysis showed that the AUC of sepsis combined with SOFA score and q-SOFA score was 0.880; the AUC of sepsis assessed by SOFA score, q-SOFA score, and △SOFA score was 0.929; the AUC of sepsis prognosis assessed by SOFA score, q-SOFA score, and △SOFA score was 0.900.

**Conclusion:**

SOFA score, q-SOFA score, and △SOFA score were abnormally expressed in patients with sepsis and were risk factors for the severity of the patient's condition and prognosis. The SOFA score, q-SOFA score, and △SOFA score were risk factors for the severity and prognosis of patients with sepsis and had some value in diagnosing sepsis and assessing the condition and prognosis, of which the combined value of the three was higher.

## 1. Introduction

Sepsis is a systemic inflammatory response syndrome caused by interference, which is a common disease in intensive care unit (ICU). Sepsis has the characteristics of high incidence rate, serious illness, rapid disease development, and high mortality and has become the focus of medical scholars all over the world [1, 2]. At present, the pathogenesis of sepsis is not completely clear, but most studies believe that the pathogenesis of sepsis is closely related to the changes of immune function and cell/organ function and the imbalance of inflammation-anti-inflammatory system. Early diagnosis and evaluation of the prognosis of patients are of great significance for early effective treatment and improving the prognosis of patients [3, 4].

Acute physiology and chronic health scoring system II (APACHE II) is a common way to evaluate the condition and prognosis of patients with acute and critical diseases in clinic, but it needs complex calculation method and long calculation time, which may affect the early effective treatment of patients [5, 6]. Sequential organ failure assessment (SOFA) is a scale widely used in emergency, internal medicine, surgery, and ICU to evaluate the disease condition and prognosis of patients with multiple organ failure, which can dynamically reflect the changes of organ function [7]. Quick sequential organ failure assessment (q-SOFA) is a scale that can quickly analyze the changes of patients' condition by analyzing consciousness, systolic blood pressure, and heart rate [8]. △SOFA score is a new quantitative index in recent years, which analyzes the changes of organ function through the fluctuation of patients' SOFA score within 24 hours.

In this study, a total of 140 patients with sepsis from January 2020 to January 2021 were selected as the objective in the present study to analyze the clinical significance of the SOFA score in the diagnosis, treatment, and prognostic assessment of sepsis.

## 2. Materials and Methods

### 2.1. General Information

140 patients with sepsis from January 2020 to January 2021 were selected as the observation group. Inclusion criteria: (1) all patients met the diagnostic criteria for sepsis published by the International Conference on Sepsis; (2) patients and their families were informed and had good compliance. They could cooperate with the examination and treatment and had signed the informed consent. Exclusion criteria: (1) patients with severe dysfunction of previous important organs; (2) patients had antibiotics and hormone therapy within 1 month; (3) the patient died or gave up the treatment within 24 hours after entering ICU; (4) the patient was complicated with blood and immune related diseases. Forty cases from the healthy population were selected as the control group. The observation group was divided into mild group, severe group, and septic shock group by single-blind grouping method according to the disease condition. Additionally, the patients were divided into the survival group and the death group according to whether they died within 28 days. The operation in this experiment was approved by the Ethics Committee of the hospital. Process of general information selection is shown in Figure 1.

### 2.2. Outcome Measures

Serum test: the morning fasting venous blood of patients with sepsis within 24 hours after admission was collected, centrifuged at 3000 r/min for 15 minutes. The supernatant was frozen in the refrigerator at -80°C to avoid repeated freezing and thawing. The levels of total bilirubin (TBIL), creatinine (CR), and platelet count (PLT) were detected by automatic biochemical analyzer. Therein, the normal range of TBlL was 5.13-22.24 *μ*mol/L; the normal range of Scr was 44-133 *μ*mol/L; the normal range of PLT was (100 − 300) × 109/L.

Scale and clinical index detection: first, a quality control (QC) team was built. The team members were composed of the ICU head nurse, the head nurse of the physical examination center, the patient responsible nurses, and the physical examination nurses. They had rich clinical experience and were proficient in relevant scales and index detection methods and had received unified training. All subjects were evaluated within 24 h of admission, including mean arterial pressure (map), partial pressure of oxygen 2/fraction of inspiration oxygen 2 (PO2/FiO2), APACHE II score, Glasgow Coma Score (GCS), SOFA score, q-SOFA score, and △SOFA score. APACHE II score [9] included the age score, acute physiology score, and chronic health status score. Scores ranged from 0 to 25 points. The higher the score was, the more serious the patient's condition was. The GCS score [10] included eye-opening movement, language response, and motor response. The score ranged from 3 to 15 points. The higher the score was, the more serious the patient's disturbance of consciousness was. SOFA score [11] was a quantitative scoring index that dynamically describes sepsis-related organ dysfunction, including respiratory system, coagulation system, liver function, cardiovascular system, central nervous system, and renal function. Scores ranged from 0 to 24 points. The higher the score was, the more serious the sepsis related organ dysfunction was. The q-SOFA score [12] included respiratory rate, consciousness change, and systolic blood pressure. Scores ranged from 0 to 3 points. The higher the score was, the more serious the organ dysfunction was. △SOFA score was the difference of SOFA score of sepsis patients before and after treatment.

### 2.3. Statistical Analysis

The experimental data were analyzed using Spss20.0 software. Age was expressed by (−*x* ± *s*). The age and other measurement data including SOFA score and △SOFA score conformed to the normal distribution and were expressed as (−*x* ± *s*). The independent samples-*t* test was used for comparison between two groups, and the SNK-q test was used for pairwise comparison of multisample means between each group. The gender and other enumeration data were expressed in (%) and compared using *χ*^2^ test. Pearson correlation analysis was used to analyze the correlation between SOFA score and other indicators. The influencing factors of patients with sepsis were analyzed by multivariate logistic regression; clinical value of SOFA score in the early diagnosis and prognosis of sepsis SOFA was analyzed through receiver-operating characteristic (ROC). *P* < 0.05 was statistically significant.

## 3. Results

### 3.1. Analysis of SOFA Score and Related Indexes of Subjects in the Two Groups

The levels of APACHE II score, SOFA score, q-SOFA score, TBIL, and Scr level in the observation group were significantly increased compared to these in control group, and the levels of MAP, PO2/FiO2, PLT level, and GCS score in the observation group were obviously decreased than these in control group (*P* < 0.05) (Table 1).

### 3.2. Comparison of SOFA Score and Related Indexes in Patients with Sepsis in Different Conditions

Apache II score, SOFA score, q-SOFA score, TBIL, and Scr levels in severe group and septic shock group were much higher than these in mild disease group, while △SOFA score, map, PO2/FiO2, PLT level, and GCS score in severe group and septic shock group were sharply lower than these in mild disease group. The levels of APACHE II score, SOFA score, q-SOFA score, TBIL, and Scr levels in the septic shock group were evidently increased compared that these in severe group, while the levels of MAP, PO2/FiO2, PLT, and GCS levels were clearly decreased relative to these in severe group (*P* < 0.05) (Table 2).

### 3.3. Comparison of SOFA Score and Related Indexes in Patients with Sepsis with Different Prognosis

The age, APACHE II score, SOFA score, q-SOFA score, TBIL, and Scr levels in the death group were strongly increased compared to these in survival group, while the △SOFA score, MAP, PO2/FiO2, PLT level, and GCS score were obviously decreased than these in survival group (*P* < 0.05) (Table 3).

### 3.4. Correlation Analysis between SOFA Score and Sepsis-Related Indexes

Pearson correlation analysis showed that SOFA score was significantly positively correlated with TBIL and Scr (*r* = 0.618, 0.479, both *P* < 0.05), and negatively correlated with MAP, PO2/FiO2, PLT and GCS score (*r* = −0.521, -0.473, all *P* < 0.05); q-SOFA score was positively correlated with TBIL and Scr (*r* = 0.571, 0.412, both *P* < 0.05), and negatively correlated with MAP, PO2/FiO2, PLT, and GCS (*r* = −0.418, -0.496, all *P* < 0.05); △SOFA score was negatively correlated with TBIL and Scr (*r* = −0.573, -0.511, *P* < 0.05), and positively correlated with MAP, PO2/FiO2, PLT, and GCS (*r* = 0.518, 0.419, all *P* < 0.05) (Table 4).

### 3.5. Analysis of Prognostic Risk Factors in Patients with Sepsis

Multivariate logistic regression analysis showed that APACHE II score, SOFA score, and q-SOFA score were independent risk factors for sepsis, and △SOFA score, PO2/FiO2, and GCS score were protective factors (*P* < 0.05) (Table 5). Nomogram analysis was shown in Figure 2.

### 3.6. Analysis of the Value of SOFA Score in the Diagnosis, Treatment Evaluation, and Prognosis of Sepsis

According to the ROC curve analysis, the AUC of SOFA score and q-SOFA score in the diagnosis of sepsis were 0.805 and 0.763, respectively, and the AUC of combined diagnosis of sepsis was 0.856; the AUC of sepsis patient's condition assessed by SOFA score, q-SOFA score, and △SOFA score were 0.759, 0.716, and 0.685, respectively, and the AUC of sepsis patients assessed by the combination of the three was 0.786; the AUC of SOFA score, q-SOFA score, and △SOFA score in evaluating the prognosis of patients with sepsis were 0.782, 0.753, and 0.714, respectively, and the AUC of the three combined in evaluating the prognosis of patients with sepsis was 0.826. (Table 6 and Figure 3).

## 4. Discussion

Sepsis is a common acute and critical disease in ICU, which is mostly seen in patients with large-area burns, severe trauma, and major surgery. Sepsis may induce acute circulatory failure and multiple organ dysfunction, which seriously threatens human life safety [13, 14]. Sepsis and septic shock are important problems faced by the Department of Critical Medicine, with high risk of death and high medical cost. Early identification and appropriate treatment can improve the prognosis of patients with sepsis, and it is of great significance to judge the severity of sepsis and guide treatment. Early identification of sepsis complicated with organ failure is particularly important, but there is still a lack of unified evaluation indicators for the risk of death and prognosis of sepsis. Therefore, it has become a hot spot in clinical research to find methods for early diagnosis of sepsis and evaluation of disease changes and prognosis.

SOFA score is a widely used quantitative index that can dynamically describe the organ function of the body. It is widely used in clinic to evaluate the multiorgan dysfunction by analyzing the respiratory oxygenation, liver function, renal function, cardiovascular system, coagulation system, and nervous system [15]. The q-SOFA score is a more rapid and simple quantitative index of ESICM/SCCM retrospective analysis, which can also evaluate the multiorgan dysfunction of the body. The advantage of q-SOFA score is that it does not need laboratory testing and is suitable for early screening and evaluation of patients in emergency and general wards. However, due to the lack of support of laboratory indicators, it may be difficult to evaluate the prognosis [16]. Some scholars used the q-SOFA score in early sepsis screening in emergency and concluded that the score can be used as a tool for early sepsis screening in emergency trauma patients [17]. △SOFA score is a method to analyze the changes of patients' organ function through the changes of patients' SOFA score within 24 hours [18]. In this experiment, there were significant differences in SOFA score, q-SOFA score, and △SOFA score of sepsis in different conditions and prognosis, suggesting that the changes of SOFA score, q-SOFA score, and △SOFA score may be helpful to diagnose and evaluate the condition and prognosis of sepsis. Observing the dynamic change trend of SOFA is helpful for the judgement of patients' prognosis, which is similar to the research from Chen et al. [19]. In addition, this study also found that there was a certain correlation between SOFA score, q-SOFA score, and △SOFA score and TBIL, Scr, PO2/FiO2, and PLT, which further confirmed the significance of SOFA score in the progression of sepsis. Liu et al. [20] discovers that the area under the ROC curve of SOFA predicting mortality is 0.890, which is higher than qSOFA. SOFA can be used as an effective auxiliary risk stratification tool for critically ill COVID-19 patients at admission, and q-SOFA is less sensitive than SOFA. Therefore, the present study believes that whether q-SOFA could be used to screen elderly patients with sepsis in China still needs to be further discussed.

Sepsis progresses rapidly, which can rapidly round into severe sepsis and septic shock with the mortality as high as 50%. Early diagnosis and evaluation of the condition is conducive to giving effective corrective treatment and reducing the mortality of patients [21]. In order to further analyze the value of SOFA score and other indicators in the diagnosis of sepsis, ROC curve analysis was carried out in the present study. It was found that SOFA score, q-SOFA score, and △SOFA score alone and in combination had certain value in the diagnosis, condition change, and prognosis evaluation of sepsis. Among them, the combined diagnostic value of the two or three index is significantly higher than that of the single index, which is helpful to help doctors make early diagnosis and give effective targeted treatment, and is of great significance to improve the prognosis of patients. Some scholars [22] demonstrate that the change of SOFA score in patients with sepsis reflected the organ function status of patients, and SOFA score shows high accuracy in describing the course of organ dysfunction in patients with severe sepsis. Big data analytics shows that q-SOFA score can also evaluate the prognosis of patients with sepsis, which can help to find sepsis and perform therapy as soon as possible. It has discovered that the q-SOFA standard performs as well or better in predicting critical diseases as the SIRS standard, severe sepsis standard, and lactate level. In this study, q-SOFA score had certain functions in predicting the diagnosis, condition, and prognosis of patients with sepsis.

In conclusion, the abnormal expression of SOFA score, q-SOFA score, and △SOFA score was a risk factor for the severity and prognosis in patients with sepsis, which had a certain value in diagnosing sepsis and evaluating the condition and prognosis. In addition, the combined value of these three indexes was higher. However, due to the limited research time and sample size, there may be some deviation in the experimental results. The sample size and research time will be expanded for in-depth exploration in our following research.

## Figures and Tables

**Figure 1:** Process of general information selection.

**Figure 2:** Nomogram analysis. Note: n-SOFA represents △SOFA.

**Figure 3:** ROC curve analysis. (a) The value of SOFA score in the diagnosis of sepsis; (b) the value of SOFA score in evaluating the changes of sepsis; (c) diagnostic value of SOFA score in prognosis of sepsis.

**Table 1:** Analysis of SOFA score and related indexes of subjects in the two groups (−*x* ± *s*).

Index	The control group (*n* = 40)	The observation group (*n* = 140)	*t/χ* ^2^	*P*
Age (year)	52.63 ± 5.96	51.96 ± 7.43	0.523	0.601
Gender (cases)				
Male	25 (62.50%)	95 (67.86%)	0.041	0.838
Female	15 (37.50%)	45 (32.14%)		
APACHE II score (score)	5.63 ± 2.15	15.52 ± 5.85	10.484	<0.001
SOFA score (score)	2.58 ± 0.16	9.18 ± 0.12	283.564	<0.001
q-SOFA score (score)	0.52 ± 0.12	1.96 ± 0.48	18.771	<0.001
MAP (mmHg)	95.23 ± 4.88	73.48 ± 3.45		
PO2/FiO2	298.63 ± 30.25	168.96 ± 35.52	21.004	<0.001
PLT (×10^9^/L)	228.63 ± 23.96	185.63 ± 22.45	10.524	<0.001
TBIL (*μ*/L)	10.26 ± 1.05	15.63 ± 2.46	13.439	<0.001
Scr (*μ*mol/L)	68.95 ± 10.26	246.96 ± 4.85	154.251	<0.001
GCS (score)	15.00 ± 0.00	9.73 ± 2.13	—	—

**Table 2:** Comparison of SOFA score and related indexes in patients with sepsis in different conditions (−*x* ± *s*).

Index	Mild disease group (*n* = 46)	Severe group (*n* = 68)	Septic shock group (*n* = 26)	*F/χ* ^2^	*P*
Age (year)	50.63 ± 5.16	52.18 ± 2.64	51.30 ± 4.16	2.200	0.114
Gender (cases)					
Male	30 (65.22%)	38 (55.88%)	17 (65.38%)	1.294	0.523
Female	16 (34.78%)	30 (44.12%)	9 (34.62%)		
APACHE II score (score)	12.08 ± 2.15	15.96 ± 3.46^a^	17.85 ± 1.62^ab^	42.400	<0.001
SOFA score (score)	6.89 ± 2.85	9.15 ± 2.46^a^	11.02 ± 2.86^ab^	21.350	<0.001
q-SOFA score (score)	1.52 ± 0.49	1.92 ± 0.29^a^	2.28 ± 0.19^ab^	40.080	<0.001
△SOFA (score)	1.39 ± 0.85	0.26 ± 0.52^a^	−2.85 ± 2.16^ab^	124.600	<0.001
PO2/FiO2	185.69 ± 10.46	167.96 ± 15.85^a^	140.63 ± 25.96^ab^	59.980	<0.001
MAP (mmHg)	88.23 ± 5.21	75.33 ± 4.26	70.15 ± 4.16		
PLT (×10^9^/L)	198.63 ± 12.64	182.63 ± 22.41^a^	139.65 ± 62.37^ab^	29.150	<0.001
TBIL (*μ*/L)	12.69 ± 2.69	15.89 ± 2.85^a^	18.06 ± 2.64^ab^	35.070	<0.001
Scr (*μ*mol/L)	208.96 ± 20.16	236.12 ± 15.23^a^	352.69 ± 26.3^ab^	488.370	<0.001
GCS (score)	12.25 ± 2.11	10.15 ± 1.26^a^	7.42 ± 1.05^ab^	80.320	<0.001

Note: ^a^*P* < 0.05 compared with the mild disease group; ^b^*P* < 0.05 compared with the severe group.

**Table 3:** Comparison of SOFA score and related indexes in patients with sepsis with different prognosis (−*x* ± *s*).

Index	The survival group (*n* = 88)	The death group (*n* = 52)	*t/χ* ^2^	*P*
Age (year)	50.46 ± 3.96	53.01 ± 4.97	3.343	<0.001
Gender (cases)				
Male	55 (62.50%)	33 (63.46%)	0.012	0.909
Female	33 (37.50%)	19 (36.54%)		
APACHE II score (score)	13.63 ± 3.85	17.98 ± 2.46	7.307	<0.001
SOFA score (score)	7.85 ± 2.46	12.05 ± 1.85	10.653	<0.001
q-SOFA score (score)	1.68 ± 0.74	2.31 ± 1.85	2.838	0.005
△SOFA score	1.05 ± 0.28	−2.56 ± 0.25	76.638	<0.001
MAP (mmHg)	80.26 ± 4.26	71.26 ± 3.25		
PO2/FiO2	190.56 ± 29.85	135.64 ± 26.38	10.972	<0.001
PLT (×10^9^/L)	186.63 ± 42.85	128.96 ± 41.36	7.793	<0.001
TBIL (*μ*/L)	13.26 ± 2.95	18.63 ± 3.10	10.191	<0.001
Scr (*μ*mol/L)	226.93 ± 20.15	361.05 ± 24.38	35.158	<0.001
GCS (score)	10.26 ± 1.25	7.05 ± 1.36	14.207	<0.001

**Table 4:** Correlation analysis between SOFA score and sepsis-related indexes.

Index		MAP	PO2/FiO2	PLT	TBIL	Scr	GCS score
SOFA score	*r*	-0.518	-0.521	-0.473	0.618	0.479	-0.426
	*P*	0.004	0.005	0.016	0.001	0.014	0.015
q-SOFA score	*r*	-0.621	-0.418	-0.496	0.571	0.412	-0.326
	*P*	0.001	0.028	0.012	0.004	0.036	0.023
△SOFA score	*r*	0.429	0.518	0.419	-0.573	-0.511	0.526
	*P*	0.008	0.006	0.035	0.004	0.008	0.002

**Table 5:** Analysis of prognostic risk factors in patients with sepsis.

Index	*Β*	SE	Wald	*P*	OR	95% CI
APACHE II score	0.289	0.076	15.234	0.001	1.325	1.145-1.562
SOFA score	0.389	0.127	10.256	0.001	1.459	1.174-1.892
q-SOFA score	0.448	0.125	3.562	0.005	1.568	1.078-1.985
△SOFA score	-0.481	0.165	9.856	0.003	0.645	1.085-2.361
MAP	-0.521	0.254	3.452	0.055	0.265	0.135~2.354
PO2/FiO2	-0.256	0.079	9.856	0.005	0.279	1.089-1.568
PLT	-0.495	0.158	2.825	0.058	0.564	1.135-2.085
TBIL	1.415	0.785	3.519	0.068	4.115	0.985-18.524
Scr	2.056	0.815	2.139	0.088	1.854	0.989-2.457
GCS score	-3.261	0.745	4.168	0.026	0.426	0.128~1.578
Age	0.005	0.006	2.541	0.102	0.985	0.941-1.025

**Table 6:** Analysis of the value of SOFA score in the diagnosis, treatment evaluation and prognosis of sepsis.

Index		AUC	95% CI	Sensitivity	Specificity	*P*
Diagnosis	SOFA score	0.767	0.759-0.861	82.64%	80.12%	<0.001
	q-SOFA score	0.796	0.718-0.801	78.63%	78.52%	<0.001
	Combined scoring	0.880	0.801-0.912	86.32%	87.14%	<0.001

Changes in the patient's condition	SOFA score	0.724	0.701-0.816	76.85%	78.45%	<0.001
	q-SOFA score	0.759	0.665-0.868	73.15%	72.58%	<0.001
	△SOFA score	0.772	0.632-0.829	70.12%	70.19%	<0.001
	Combined scoring	0.929	0.724-0.829	89.52%	90.12%	<0.001

Prognosis	SOFA score	0.755	0.655-0.825	79.52%	81.66%	<0.001
	q-SOFA score	0.763	0.669-0.819	78.44%	79.52%	<0.001
	△SOFA score	0.756	0.660-0.764	72.64%	75.21%	<0.001
	Combined scoring	0.900	0.841-0.960	85.49%	82.67%	<0.001

## Data Availability

The datasets used and/or analyzed during the current study are available from the corresponding author on reasonable request.
